This article has been retracted.

# Research on Diagnosis Architecture of Cardiovascular Diseases Based on Multimedical Images

**DOI:** 10.1155/2022/9123332

**Published:** 2022-02-09

**Authors:** Chunying Yu, Yani Che, Guifang Sun, Xipeng Zhao, Bin Liu

**Affiliations:** ^1^Radiology Department, Shaanxi Normal University Hospital, Xi'an, Shaanxi 710062, China; ^2^Radiophysics Department, Qingdao Central Hospital, Qingdao, Shandong 266042, China; ^3^Radiology Department, Yan'an Hospital of Kunming City, Kunming, Yunnan 650051, China; ^4^Molecular Imaging Department, Qingdao Central Hospital, Qingdao, Shandong 266042, China

## Abstract

**Objective:**

To study the effect of a multi-image source 3D modeling imaging examination system on the diagnosis of cardiovascular diseases in cardiac surgery.

**Methods:**

The data of 680 confirmed patients and 1590 suspected patients in the cardiac surgery department of all hospitals of a large chain hospital management group were selected. All patients gave the examination results of multiple image sources and independent examination results of multiple image sources, respectively, their examination sensitivity, specificity, and reliability were compared, and the treatment efficiency and nursing satisfaction of the virtual reference group were deduced in MATLAB. Perform the bivariate *t*-test and comparative statistics in SPSS.

**Results:**

The multi-image source 3D modeling examination system had higher examination sensitivity, specificity, and reliability and higher examination sensitivity in the early stage of the disease. It was deduced that the clinical efficiency and nursing satisfaction based on the examination results were significantly improved (*t* < 10.000, *p* < 0.01).

**Conclusion:**

The multi-image source 3D modeling imaging examination system is suitable for the diagnosis of cardiovascular diseases in cardiac surgery.

## 1. Introduction

The cardiovascular system includes two sets of the circulatory system: one is the three branches of the coronary artery supplying the heart itself and the myocardial supporting capillary system and the other is the aorta, pulmonary artery, superior vena cava, inferior vena, cava and pulmonary vein system supplying systemic blood circulation [1]. The latter is called the cardiac macrovascular system, which mainly investigates the complex connection structure and valve structure between macrovessels [2]. The cardiovascular system is also called the “circulatory system.” It is composed of the heart, artery, capillary, and vein. It is a closed circulation pipeline in which blood flows, supplies oxygen, various nutrients, and hormones to organs and tissues, and transports the waste of tissue metabolism to the excretory organs, so as to maintain the homeostasis of the internal environment and the progress of metabolism and maintain normal life activities. The system consists of the heart, arteries, capillaries, veins, and blood flowing therein [3]. The heart can automatically and rhythmically contract and relax under the control of the nervous system to ensure the circulation of blood in a certain direction. Arteries connect between the heart and capillaries and carry blood from the heart to tissues. Capillaries are connected between arteries and veins and form a network. They are the sites of material exchange between blood and tissues. Veins connect between capillaries and the heart, collecting blood and flowing back to the heart [4].

Common cardiovascular diseases include aortic dissection, vasculitis, arteriosclerosis, valve murmur (mitral valve, tricuspid valve, aortic valve, and pulmonary valve), etc. The root cause is the change of biological structure and mechanical properties of large blood vessels and even the change of structural strength, resulting in the change of blood flow signal and ECG signal. Due to the continuous movement of the heart, the imaging effects of MRI, MRA, and X-ray tomography based on solid imaging in the surrounding area of the heart are poor. Therefore, at present, hospitals tend to use Doppler imaging and electronic tomography for enhanced scanning imaging and form a three-dimensional model for clinical evaluation [5]. Long-term hypertension can thicken or harden the arterial wall, narrow the lumen, and then affect the blood supply to the heart and brain. Hypertension can aggravate the heart load, be prone to left ventricular hypertrophy, and further lead to hypertensive heart disease and heart failure. When blood pressure rises suddenly, cerebral vessels are easy to rupture and intracerebral hemorrhage occurs; the hardened cerebral arterioles form a chestnut-sized microaneurysm, which ruptures when the blood fluctuates, resulting in intracerebral hemorrhage; hypertension accelerates the process of arteriosclerosis; arterial endothelial cells are damaged; platelets are easy to accumulate in the injury; and it is easy to form thrombosis, leading to myocardial infarction or cerebral infarction [6].

This study focuses on the overall analysis of the new image management technology in the process of imaging diagnosis of cardiovascular diseases in the hospital and analyzes the impact of the new model on the sensitivity, specificity, and reliability of diagnosis from the perspectives of image big data management and diagnosis process management. Medical image diagnosis occupies a considerable proportion in modern medical activities. With the continuous development of visualization technology, modern medicine is increasingly inseparable from the information of medical images, which is playing an extremely important role in clinical diagnosis and medical research. Medical image information is diversified, such as B-ultrasound scanning image, color Doppler ultrasound image, nuclear magnetic resonance image, X-CT image, and X-ray fluoroscopy image. With the in-depth development of medical diagnosis visualization technology, people are making continuous efforts to seek clearer and more diagnostic value of high-quality medical images.

## 2. New Image Diagnosis Management Process and Medical, Technical, and Nursing Cooperation Mode

Internet plus health mode is an important form of social development in China in recent years and its application in the medical industry. Its performance exists not only in the cooperation mode between hospital institutions and patients, family members, and other service providers but also in the cooperation mode between various departments and staff within the hospital. In Internet plus health mode, there is a significant change in the cooperation mode between medical, technical, and nursing personnel in hospital and the cooperation mode of medical, technical, and nursing care in traditional western medicine hospitals, as shown in Figure 1. Note that the Internet plus is the further practice of Internet thinking, which promotes the continuous evolution of the economic form, thereby promoting the vitality of the social economic entities and providing a broad network platform for reform, innovation, and development. Popularly speaking, Internet plus is the “Internet plus all traditional industries,” but this is not simply a combination of the two. It is the use of information and communication technology and the Internet platform to enable the Internet to merge with traditional industries in depth and create new development ecology. It represents a new social form, that is, giving full play to the optimization and integration role of the Internet in the allocation of social resources, deeply integrating the innovative achievements of the Internet into all economic and social fields, and improving the innovation and productivity of the whole society.

In Figure 1, according to the general examination results of surgery, the cardiac surgeon issues relevant checklists. Under the management of the nursing department on patients and examination results, the imaging doctor performs the examination process and finally generates a three-dimensional model according to the comprehensive examination results. At this time, the imaging doctor will give preliminary examination opinions according to the three-dimensional model, and the final diagnosis result will be given by the cardiac surgeon. Compared with the management mode of traditional modern western medical institutions, the biggest difference between the traditional mode and the above mode is that under the traditional mode, imaging doctors will give preliminary examination opinions according to each examination result, some new imaging examination processes will be assisted by computer artificial intelligence to give preliminary examination opinions, and the traditional mode does not include the three-dimensional modeling process based on multiple image sources.

The three-dimensional modeling imaging examination result is an examination result oriented to the anatomical structure. The cardiac surgeon will form cross sections from various angles according to the lesion structure and physiological anatomical structure in the three-dimensional model, measure the data, and finally obtain the diagnosis result through consultation and analysis. This model has positive significance for the early examination of the course of disease. For example, in the early stage of the course of aortic dissection, the dissection effusion is not significant, only manifesting as aortic turbulence murmur and changes in the anatomical structure of the aortic wall. It is difficult to find related lesions in the traditional mode, but it is easier to find in this mode. The Internet plus health management mode pays attention to the detailed division of labor and deep coordination of medical and technical staff in the cardiovascular surgery department. The imaging doctors have the ability to operate the imaging equipment and the ability to handle big data, and the cardiac surgeons have specialized knowledge and clinical experience in pathology, physiology, and anatomy, and the nursing staff introduce new patients and equipment. The checklist management system provides management system guarantee, and the close cooperation of the three can provide more refined cardiovascular examination operation.

For the complex and high-precision geometric shapes often faced in the industry and other fields, the geometric model definition language cannot correctly and completely describe the samples. Therefore, people gradually tend to use CAD software to assist in the geometric modeling of samples. The CAD sample model can describe very complex 3D entities and can quickly and accurately generate the surface triangular patch mesh model of the sample. The application of the CAD model in CT simulation greatly improves the application level of CT simulation, and it is also the development direction of sample modeling.

## 3. New Big Blood Vessel Big Data Management System and Artificial Intelligence Analysis System Based on Multiple Image Sources

The multisource image mentioned in this study refers to the cardiac Doppler color ultrasound and high-speed electronic spiral CT tomography for the purpose of cardiovascular surgical imaging examination, as well as the cardiac MRI and MRA examination carried out in conjunction with the above two examinations. Some patients will undergo mediated angiography based on the inferior vena cava. The three-dimensional model is generated from the above data through the three-dimensional modeling software. The cardiac surgeon will perform various angle projection and slice analyses on the three-dimensional model, measure the physiological and pathological anatomical structure, measure the area of the lesion that can be clearly diagnosed, and finally form the diagnosis result. The data flow diagram of imaging big data processing is shown in Figure 2. The efficient image fusion method can comprehensively process the information of multisource channels according to the needs, so as to effectively improve the utilization of image information, the reliability of target detection and recognition, and the degree of automation of the system. Its purpose is to synthesize the multiband information of a single sensor or the information provided by different sensors and eliminate the possible redundancy and contradiction between multisensor information, so as to enhance the information transparency in the image, improve the accuracy, reliability, and utilization rate of the interpretation, and form a clear, complete, and accurate information description of the target.

In Figure 2, from the perspective of the medical examination technology department, a three-dimensional modeling and analysis system is installed at the back end of the imaging examination equipment, and all data analysis functions are integrated into the system assembly. The research does not involve the software and hardware development tasks of relevant equipment. However, from the perspective of nursing management, the system needs the support of auxiliary systems such as electronic medical record system and online consultation system, and the examination equipment needs the preliminary three-dimensional model data export function; that is, the Doppler ultrasound equipment and electronic spiral CT equipment purchased earlier need to add a three-dimensional model data export module. From the perspective of nursing management, the system upgrade objectives are shown in Figure 3. In addition, three-dimensional imaging refers to the method of presenting two images with potential difference to the left and right eyes of the observer, respectively. It constructs or enhances the visual depth of the image by combining the two-dimensional images in the observer's brain to form a three-dimensional depth.

In Figure 3, from the perspective of the three service departments of medicine, technology, and nursing, the introduction of the system will involve the following innovations. (1) From the perspective of the imaging technology department, the imaging equipment is upgraded and transformed, and the preliminary 3D model building function module and the inspection result 3D model data export module are added. This module will be directly connected with the electronic medical record system, and the data can be imported into the overall imaging inspection result 3D modeling equipment to generate the overall layered 3D model. The 3D model modeling result data will also be imported into the electronic medical record system. (2) From the perspective of the clinical department of cardiac surgery, the final diagnosis result notice and relevant doctor's orders were prepared by viewing the examination result documents of the imaging department in the early stage and relying on clinical experience. After the innovation, the three-dimensional model of the patient's heart and surrounding regional tissues provided by the online consultation system can be used to simulate physiological anatomy and pathological anatomy, and the computer artificial intelligence-aided diagnosis tool provided by the three-dimensional modeling system can be used to obtain a more objective notice of diagnosis results, so as to provide computer-aided functions for the accuracy, objectivity, and reliability of medical orders. (3) According to the nursing manual, the three major tasks of nursing work include the following: patient diagnosis and treatment channel management (medical guidance, inspection equipment, and ward management), patient medical record file management, and medical order execution and nursing operation process management. After the deployment of the multisource image diagnosis and treatment system, the workload of patient medical record file management in nursing work has increased significantly. Nurses should ensure the data reliability of the electronic medical record system and online consultation system and promote all departments to upload data in time according to regulations. In the management of the patient diagnosis and treatment channel, it is necessary to ensure that each examination time window of patients is timely and reasonable, so as to avoid the distortion of patient examination results caused by unreasonable imaging examination sequence and examination time. For example, in patients with aortic dissection, the examination time interval may be 1 hour, and the imaging results of the two examinations will be significantly different, resulting in the distortion of the three-dimensional model data. The 3D model itself is invisible. It can be rendered at different levels of detail according to a simple wireframe or painted in different ways. However, many 3D models use texture to overlay, and the process of arranging the texture on the 3D model is called texture mapping. Texture is an image, but it can make the model more detailed and look more realistic.

## 4. Clinical and Nursing Value Research Scheme of the Multi-Image Source Examination System

### 4.1. Clinical Data of Patients

A chain hospital management group governs 24 third-class general hospitals and 65 second-class general hospitals. All hospital institutions have set up cardiovascular surgery departments and provide outpatient and inpatient diagnosis and treatment services, and all hospitals receive patients from cardiovascular surgery. 680 patients with cardiovascular diseases treated by the hospital management group in 2020 were selected, including the following: (1) 240 patients with aortic dissection, aged 33-72 years, with an average of 54.6 ± 2.7 years, 186 males and 54 females, with a diastolic blood pressure of 160~193 mmHg, an average diastolic blood pressure of 177.6 ± 24.5 mmHg, a course of hypertension of 0.2~3.5 years, and an average course of 1.32 ± 0.18 years; (2) 380 patients with macrovascular atherosclerosis, aged 36~73 years, with an average of 53.7 ± 5.3 years, 266 males and 114 females, with the performance of hyperlipidemia (calculated by serum triglyceride) being 4.9~9.2 mmol/l and the average performance of hyperlipidemia being 7.41 ± 0.92 mmol/l and the course of hyperlipidemia being 2.2~6.5 years, with an average course of 3.45 ± 0.72 years; and (3) 210 patients with secondary degenerative valve murmur, aged 47~81 years, with an average age of 62.7 ± 4.1 years. There were 72 males and 138 females, with a course of 0.4 ~ 4.5 years and an average course of 1.22 ± 0.28 years. Among the above patients, 150 patients with cardiovascular disease complications were investigated, and all patients had symptoms of hypertension, hyperglycemia, and hyperlipidemia. Patients with renal dysfunction such as hyperuricemia and hyperketosis were excluded from the study, and some patients were complicated with coronary atherosclerosis. The image of coronary atherosclerosis was not considered in the study. However, patients with myocardial infarction and its sequelae were excluded from the study. All patients had not undergone cardiac surgery before seeing a doctor.

### 4.2. Imaging Examination Plan and Cardiac Surgery Treatment Plan

The study focused on the impact of multisource imaging on the sensitivity, specificity, and reliability of the examination and the impact of multisource imaging on the surgical results and nursing satisfaction. Therefore, the surgical schemes of all patients were the same. The following surgical treatment schemes were selected according to the actual conditions of the patients: (1) aortic dissection and restoration or artificial vascular replacement was performed in patients with aortic dissection, (2) patients with aortic atherosclerosis underwent aortic stent implantation or artificial vascular replacement, and (3) patients with valve murmur underwent valve correction or artificial valve replacement. The nursing management system adopts the whole person nursing path facing the whole life cycle.

In the patient statistics, after completing the medical record screening and drop statistics, the above 680 patients were confirmed patients. At the same time, the follow-up results of 1590 suspected patients were investigated, and the missed patients under the specific influence of statistical examination were counted. That is, the examination process of all patients is divided into two steps. The clinical practice is to implement the examination scheme based on multiple image sources involved in the study. In addition, the examination results based on separate imaging examinations are simulated, and the operation process is deduced as the reference group. The research model takes into account the impact of medical ethics; that is, it has been convinced theoretically that multisource imaging can provide high examination sensitivity, specificity, and reliability. It is strictly prohibited to implement other examination schemes that are clearly detrimental to the patient's health and life safety. The specific statistical results will be discussed below. After the reasonable selection of data, it is necessary to preprocess it first, so as not to affect the fusion effect of unprocessed data in multisource fusion. The method of data preprocessing mainly includes geometric calibration of various selected data signals and images and then conversion of all data into image format. Preprocessing must ensure that all data can communicate with each other and that data fusion can be realized on the same platform.

### 4.3. Statistical Methods of Clinical and Nursing Data

Count data counts the total number of samples, effective data count result *N*, and the proportion of effective data in the total number of samples *A*%, which is displayed in the statistical results in the format of *N* (*A*). The mean value *X* of measurement data statistics (statistical method such as formula (1)) and standard deviation rate *S* (statistical method such as formula (2)) and the statistical results are displayed in the results in the format of *X* ± *S*.

The mean value calculation method of formula (1) is the arithmetic mean measurement method:

(1) $$\begin{array}{c} A=\frac{1}{n}\overset{n}{\underset{i=1}{\sum }}\lambda_{i}\cdot T_{i}, \end{array}$$

where *T*_*i*_ is the *i*-th statistical input value; *λ*_*i*_ is the weight of the *i*-th statistical input value, which is equal to 1 without special statistical requirements; *n* is the total number of samples; and *A* is the arithmetic average output result.

The calculation method of the standard deviation rate in formula (2) is a factor-enhanced standard deviation rate calculation scheme:

(2) $$\begin{array}{c} S=\sqrt{\frac{1}{n-1}\overset{n}{\underset{i=1}{\sum }}{\left(T_{i}-A\right)}^{2}}, \end{array}$$

where *T*_*i*_ is the *i*-th statistical input value, *A* is the arithmetic mean of all statistical input values (see formula (1) for details), *N* is the number of statistical samples, and *S* is the statistical result of the standard deviation rate.

Besides, standard deviation is the most commonly used quantitative form to reflect the dispersion of a group of data. It is an important indicator of accuracy. Although it is impossible to know the true value of the sample, each sample will always have a true value, no matter how much it is. It is conceivable that the detection value of a good detection method should be closely scattered around the real value. If it is not close, the distance from the real value will be large and the accuracy will certainly be poor. It is impossible to imagine a method with large dispersion to measure accurate results. Therefore, dispersion is the most important and basic index to evaluate the quality of the method.

The data difference comparison scheme adopts the bivariate *t*-check method based on an SPSS big data analysis tool. The value value and log value are read from the bivariate *t*-check output results, in which the value value is displayed as *t* value in the results. When *t* < 10.000, it is considered that there is a statistical difference in the data, and in other cases, it is considered that there is no statistical difference in the data. The log value is shown as *p* value. When *p* < 0.05, it is considered that the comparison result is within the confidence range; when *p* < 0.01, it is considered that the comparison result has significant statistical significance; and when *p* ≥ 0.05, it is considered that the comparison result has no statistical significance. The bivariate *t*-check statistical process is the packaging function of SPSS statistical tool software, which is limited by space. Its statistical formula will not be discussed here.

## 5. Clinical and Nursing Value of the Multi-Image Source Examination System

### 5.1. Sensitivity, Specificity, and Reliability of Multisource Imaging

By comparing the multisource examination mode and the mode of independent diagnosis using different image sources and comparing the statistical results of clinical data with sensitivity, specificity and reliability, Table 1 is obtained.

In Table 1, sensitivity refers to the proportion of true positive data in all positive data, sensitivity refers to the proportion of true negative data in all negative data, and reliability refers to the detection rate of true positive data. In all the comparative data of the three common cardiovascular diseases investigated in this study, there were statistical results of *t* < 10.000 and *p* < 0.01; that is, all the data had significant statistical differences.

Because the examination sensitivity of all data in patients with the early disease course and low age group has more clinical value, early intervention can effectively improve the clinical efficiency and improve the quality of life of patients. Therefore, this study especially studied the sensitivity data in the early stage of the disease course, in which the early stage of aortic dissection refers to the stage of the disease course in which the patient has aortic dissection but no significant aortic dissection effusion, and the aortic atherosclerosis and heart valve murmur in patients refer to the stage in which the patient only has palpitations, dizziness, and other atypical symptoms; Doppler examination and ECG examination cannot give the course stage of typical manifestations. The data of the early and late course of the disease are shown in Figure 4.

In Figure 4, compared with the traditional mode of making independent diagnosis based on multiple image sources, the sensitivity difference in the late stage of the disease course is small, but the sensitivity difference in the early stage of the disease course is significant; that is, the multi-image source examination mode has greater value for the sensitivity of the early stage of the disease course.

### 5.2. Subjective Evaluation of Doctors and Nursing Satisfaction of Patients

All hospitals under the hospital management group have cardiac surgery and imaging departments. There are 225 cardiac surgeons related to the study and 293 imaging doctors related to the study. The above doctors are required to make subjective evaluation on multiple problems related to the multisource examination system, with a maximum of 10 points and a minimum of 0 point. The statistical results are shown in Table 2.

In Table 2, both imaging doctors and cardiac surgeons subjectively believe that the diagnosis difficulty of the multisource imaging system is low and the system is easy to use. There are significant statistical differences in all comparative data (*t* < 10.000 and *p* < 0.01).

The treatment effectiveness and patient care satisfaction of the independent diagnosis scheme using multiple image sources are deduced to obtain the reference group. The deduction tools are the random event engine and social simulation engine under the MATLAB big data analysis platform. At the same time, the treatment effectiveness and patient care satisfaction under the three-dimensional modeling and diagnosis mode using multiple image sources are counted, and Table 3 is obtained.

In Table 3, the clinical effective rate refers to the proportion of patients who meet the clinical effective criteria in the total number of patients according to the diagnostic criteria of cardiac surgery. The surgical accident rate refers to the proportion of the number of patients who have to change to the surgical scheme or the need for secondary surgery in the total number of patients. Nursing satisfaction refers to the proportion of patients who are “satisfied” or “basically satisfied” with the hospital service level during hospitalization in the discharge evaluation survey in the total number of patients. Because there are no patients with clinical deterioration or death due to surgical accidents in this study, this scenario is not set in the deduction, so no data evaluation is given to patients with deterioration or death.

## 6. Summary

The core innovation of this research is to add 3D data modeling equipment based on multiple image sources to the data logic architecture of cardiovascular examination-related equipment in cardiac surgery and apply the 3D data modeling results given by the equipment to the electronic medical record system and online consultation system, in order to increase the diagnostic accuracy of cardiovascular-related diseases in cardiac surgery (sensitivity, specificity, and reliability). The study found that the three-dimensional data modeling equipment effectively improved the accuracy of cardiovascular examination in cardiac surgery and promoted clinical efficacy and nursing satisfaction. The weakness of the study was that subject to the ethical requirements of medical research, the objective reference group was not set up, but the virtual reference group was set up by MATLAB deduction. The study confirmed the three-dimensional data modeling for cardiovascular surgery. The equipment is helpful to improve the effect of cardiovascular surgical examination and surgical clinic.

## Figures and Tables

**Figure 1:** Execution process of multi-image source inspection.

**Figure 2:** Data flow diagram of multi-image source cardiac surgery examination results of 3D modeling big data analysis.

**Figure 3:** Upgrade target of the hospital diagnosis and treatment big data system for cardiovascular imaging examination in cardiac surgery.

**Figure 4:** Sensitivity distribution under different course conditions.

**Table 1:** Comparison of sensitivity, specificity, and reliability of two inspection modes.

Comparison items		Sensitivity	Specificity	Reliability
Aortic dissection	Multiple image sources	91.60%	87.78%	92.54%
	Separate image source	69.85%	66.67%	71.37%
	*t*	3.187	2.274	3.157
	*p*	0.003	0.005	0.004

Aortic atherosclerosis	Multiple image sources	93.83%	94.44%	95.27%
	Separate image source	87.41%	89.29%	88.62%
	*t*	6.501	5.498	5.826
	*p*	0.007	0.006	0.006

Heart valve murmur	Multiple image sources	95.02%	95.60%	95.42%
	Separate image source	89.59%	91.22%	90.54%
	*t*	7.415	9.056	8.275
	*p*	0.006	0.008	0.007

**Table 2:** Comparison of doctors' subjective evaluation related to the study.

Comparison items	Cardiac surgeon		Imaging doctor	
	Diagnostic difficulty	System ease of use	Diagnostic difficulty	System ease of use
Multiple image sources	5.3 ± 0.8	8.2 ± 1.8	4.5 ± 0.6	8.4 ± 1.5
Separate image sources	6.4 ± 0.5	7.8 ± 0.7	7.2 ± 1.3	7.5 ± 1.1
*t*	4.225	3.179	2.053	3.862
*p*	0.005	0.003	0.003	0.004

**Table 3:** Investigation and deduction results of clinical efficiency and patient satisfaction (*n* = 680).

Comparison items	Clinical effective rate	Surgical accident rate	Nursing satisfaction
Multiple image sources	654 (96.2)	11 (1.6)	632 (92.9)
Separate image sources	593 (87.2)	17 (2.5)	554 (81.5)
*t*	3.551	2.194	2.983
*p*	0.005	0.003	0.006

## Data Availability

The data underlying the results presented in the study are available within the manuscript.
